# The Alleviative Effect of Vitamin B_2_ on Potassium Bromate-Induced Hepatotoxicity in Male Rats

**DOI:** 10.1155/2020/8274261

**Published:** 2020-07-30

**Authors:** Iftekhar Hassan, Hossam Ebaid, Ibrahim M. Alhazza, Jameel Al-Tamimi

**Affiliations:** Department of Zoology, College of Science, King Saud University, Riyadh, Saudi Arabia 11451

## Abstract

Potassium bromate (PB) is a food enhancer, water disinfection by-product, and a proven carcinogen. It elicits toxicities in the living organism due to exposure and in a dose-dependent manner. The present study discourses the ameliorative efficacy of riboflavin (RF) in PB-administered rodents. The animals were distributed into five treatment groups: control (group I), PB alone (group II, 150 mg/kg), RF alone (group III, 2 mg/kg), PB+RF1 (group IV, 150 mg/kg + 2 mg/kg), and PB+RF2 (group V, 150 mg/kg + 4 mg/kg). After the round of the treatment, the animals were sacrificed to collect their blood and liver samples for the detailed analysis. Group II depicted perturbed liver functions evidenced by altered serum and toxicity markers along with the disturbed redox balance. Also, these biochemical results were found harmonious with histopathological analysis and comet assay. However, group III showed no noticeable alteration in the same parameters, whereas the combination groups (IV and V) exhibited dose-dependent amelioration in the PB-induced toxicities. Interestingly, RF favored apoptosis concomitant with suppressing the necrosis in the PB-challenged groups, as shown by the activity of caspase-3 and lactate dehydrogenase. Histopathological analysis and comet assay further consolidate these results. Hence, RF has significant alleviative property against PB-induced hepatotoxicity in vivo that can be used in the consumer items containing the toxicant.

## 1. Introduction

The exposure of humankind to the xenobiotics always poses unknown and undefined biological interactions. Many of them might be deleterious in the living system posing as a significant clinical challenge among contemporary scientists. Potassium bromate (PB) is a common food processing agent besides being used in the production of various cosmetic and pharmaceutical items since its approval for such usage. Its traces can be cited in multiple packaged and municipality supply water after ozonization during the filtration process [1]. Also, it is used in improving flour quality and dough conditioning in the baking industry as well as in the preparation of beverages, cheese, and fish paste [2–4]. Hence, PB in various consumer items poses mild to severe toxicity to critical organs, viz., the kidney, liver, and brain in the living systems [5–7]. It has been categorized as a potential class II B carcinogen for humans (IARC, 1999), while it is a confirmed carcinogen in the experimental animals attributed to its extensive oxidizing property and mutagenicity [7]. For these harmful effects, its usage in food products is banned in many countries of the European Union, Canada, and many south American, African, and Asian countries, including India, China, and Sri Lanka, yet it is used in countries like the USA and Japan with certain limitations. Also, it is restrictively or illegally used in many other countries. Various studies show that PB is a strong oxidizing agent that generates free radicals during xenobiotic metabolism. It perturbs the redox balance in the cells damaging the structural and functional status of the target tissues and macromolecules. Such derogatory effect, if prolonged, can cause many diseases, including cancer, depending on the dose, duration, and concurrent circumstances in the exposed organisms [2, 3, 7].

Vitamin B_2_ (riboflavin, RF) is a hydrosoluble vitamin. It is an essential vitamin for its role as an intermediary in the metabolism of crucial macromolecules in all living things. It occurs in the two coenzymatic forms—flavin adenine dinucleotide (FAD) and flavin adenine mononucleotide (FMN) in biological systems. These flavin proteins participate in almost 100 types of metabolic redox reactions related to stress response, body development, DNA repair, circadian rhythm, photosensitization, and activation of many vitamins, including folate and pyridoxine in all forms of life [8, 9]. Prolonged deficiency of this vitamin is rare in humans; however, its inadequacy is manifested by anemia, dermal lesions, altered metabolism, and peripheral neuropathy in the late stages. The vitamin can exert a positive or negative effect on several biologically relevant molecules, drugs, and medicines attributed to its antioxidant and photosensitizing (prooxidant) activities [10–12]. This dual property of the vitamin widens its therapeutic window under ribophototherapy and photodynamic therapy. It has been employed in killing tumors, inactivation of toxins, treatment of hyperbilirubinemia, blue nevi, skin lesions, and sterilization of blood products [13–15]. The current investigation was aimed at investigating the efficacy of RF to improve PB-induced toxic insults in male rats.

### 1.1. Hypothesis

The supplementation of vitamin B_2_ can protect from the PB-induced hepatotoxicity in rodents in a dose-dependent manner.

## 2. Materials and Methods

### 2.1. Materials

All the chemicals and reagents were procured either from Sigma Aldrich (St. Louis, MO, USA) or Biolab (UK) and Millipore Merck (Darmstadt, Germany). Most of the kits for biochemical assays and estimations used were bought from Química Clínica Aplicada diagnostic kits (Spain). The caspase-3 assay kit was procured from Thermo Fisher Scientific (USA).

#### 2.1.1. Methods

*(1) Rearing of Rats and Their Treatment*. Thirty healthy Swiss albino rats (male, 120 ± 20 g, eight weeks old) were purchased from the Central Animal House (College of Pharmacy, King Saud University (KSU), Riyadh). They were homed in specially designed commercial plastic animal cages with a controlled condition (22 ± 3°C; 72–77% relative humidity; 12 h day/night cycle) in the Departmental Animal House (Department of Zoology, KSU, Riyadh) on rat pellet diet and fresh tap water ad libitum. The rodents were divided randomly into the five groups: group I (vehicle control treated with saline), group II (potassium bromate at 150 mg/kg body weight as a single dose; [16]), group III (vitamin B_2_ at the dose of 2 mg/kg body weight twice a week for a month), group IV (a single dose of potassium bromate at 150 mg/kg body weight followed by vitamin B_2_ at the dose of 2 mg/kg body weight twice a week for a month), and group V (a single dose of potassium bromate at 150 mg/kg body weight followed by vitamin B_2_ at the dose of 4 mg/kg body weight twice a week for a month). All the test chemicals were administered intraperitoneally in the present work. The animals were killed on the same day after the completion of the treatment for sample collection. The study was approved by the Departmental Ethical Committee (Department of Zoology, KSU).

#### 2.1.2. Preparation of Samples

The animals were sacrificed for liver samples were collected after thoroughly washing with chilled phosphate-buffered saline (PBS). Then, the samples were homogenized (Ika-Werke, Germany) in Tris-KCl buffer (pH 7.36). Their supernatants were kept at −80°C with proper labeling until further analysis. Besides, the blood was also collected [17] in vacuum polystyrene collecting tubes (Corning, USA). The serum was retrieved after centrifugation (Eppendorf, Germany) at 1000 × g and was stored in the refrigerator. Apart from this, half of the liver from each animal was saved for the comet assay and histopathological study.

#### 2.1.3. Assessment of Liver Function Markers

The assay of aspartate transaminase (AST) and alanine transaminase (ALT) was carried out by the commercial kits (Química Clínica Aplicada diagnostic kits, Spain) according to the manufacturer's instructions.

#### 2.1.4. Assessment of Toxic Insult on the Liver

Gamma-glutamyl transferase (GGT), glutamyl S-transferase (GST), and thioredoxin reductase (TR) were measured in the liver samples by the commercial kits (Quimica Clinica Aplicada S.A., Spain) according to the manufacturer's manual.

#### 2.1.5. Assessment of Activity of Antioxidant Enzymes

The assay of critical antioxidant enzymes like superoxide dismutase (SOD), catalase (CAT), and glutathione reductase (GR) was done by the established protocols [18–21].

#### 2.1.6. Measurement of Reduced Glutathione (GSH) Level

The total reduced glutathione (GSH) was estimated by the method of Jollow et al. [22].

#### 2.1.7. Assessment of Macromolecular Oxidation of Lipids and Proteins

The oxidative damage to the lipids and protein was conducted by measuring the level of MDA and the carbonyl content, respectively. They were estimated by the standard protocols of Beuge and Aust (1978) and Levine et al. [23], respectively.

#### 2.1.8. Assessment of Mode of Cell Death

Commercially available kits were used for measurement of the mode of cell death in the target organs following the manufacturer's instructions (Quimica Clinica Aplicada S.A., Spain; Thermo Fisher Scientific, USA). Caspase-3 was chosen to assess the extent of apoptosis [24], whereas lactate dehydrogenase was measured for assessment of necrosis [25] in the tissue samples.

#### 2.1.9. Comet Assay of Liver Samples

The assay was done by the standard protocol of Singh et al. [26] in alkaline conditions with slight modifications [27] in the present study.

#### 2.1.10. Histopathological Assessment of Liver Tissue Samples

The fresh tissue samples were stored in an 8% formaldehyde solution in phosphate-buffered saline (PBS) after washing in PBS and dehydration in a series of alcohol dilutions and embedded in paraffin. Microtome sections were cut and adhered to slides before staining with hematoxylin and eosin. The histopathological alteration in the sections of hepatic tissue was examined blindfolded using a Leica DMRB/E light microscope (Heerbrugg, Switzerland) with an attached HD camera (Leica MC 170 HD, Singapore). Photomicrographs of the sections were taken, which were digitized using Adobe Photoshop (Adobe Systems, Mountain View, CA). All the histopathological alterations were scored as per the method of Dommels et al. [28]. A rating score of histological alteration between – (no change) and +++ (severe damage) was assigned for each section.

#### 2.1.11. Statistical Analysis

All the data has been expressed in the mean ± SD analyzed by GraphPad Prism 5 software. The data were subjected to one-way ANOVA analysis with Tukey's post hoc multiple comparison test. *p* value < 0.05 was chosen as statistically significant in the present study. The marks “a, b, and c” were used as asterisk marks to show significance difference from the negative control (CN^−^, group I) at *p* less than 0.05, 0.005, and 0.001 while the marks “x, y, and z” were used as asterisk marks to show significance difference from the positive control (CN^+^, group II) at *p* less than 0.05, 0.005, and 0.001.

## 3. Results

### 3.1. Effect on Liver Function Markers

#### 3.1.1. Alkaline Phosphatase (ALP)

ALP is a critical enzyme to assess liver functionality in vivo. Groups II and III demonstrated an increase in its activity by 419.74% and 42% as compared to the control, group I. However, treatment with riboflavin decreased its activity by 28% and 49.24% as evidenced by groups IV and V, respectively (Figure 1).

#### 3.1.2. Aspartate Transaminase (AST)

It is also considered as a significant liver function marker in in vivo studies. In the present investigation, groups II and III showed elevation of its activity by 723.01% and 282.54% concerning the control while groups IV and V displayed a decline in its activity by 24.50% and 42.03% as compared to group II (Figure 1).

#### 3.1.3. Alanine Transaminase (ALT)

Groups II and III exhibited the enhanced activity of this enzyme by 634.46% and 41%, while the combination groups IV and V showed a dip in its activity by 40.84% and 59.72%, respectively (Figure 1).

### 3.2. Assessment of Toxic Burden In Vivo

These are the prominent markers to assess the extent of the toxic load on the living system after the administration of any toxic or xenobiotic substance.

#### 3.2.1. Glutathione-S-Transferase (GST)

Groups II and III showed an elevation in its activity by 220.39% and 35.84% to the control while the combination groups IV and V exhibited a decline in its activity by 40.36% and 53.53% as compared to group II (Figure 2).

#### 3.2.2. Thioredoxin Reductase (TR)

The activity of TR was found depressed by 261.91% and 70.94% with respect to group I (control). In contrast, groups IV and V demonstrated the decline in its activity by 26.43% and 41% as compared to group II, respectively (Figure 2).

#### 3.2.3. Gamma-Glutamyl Transferase (GGT)

Groups II and III showed enhancement in its activity by 448.23% and 32.62% with respect to the control. In comparison, the combination groups IV and V exhibited a decline in its activity by 67.26% and 74.12% as compared to group II (Figure 2).

### 3.3. Effect on Antioxidative Enzymes

#### 3.3.1. Catalase (CAT)

It is a critical antioxidant enzyme in living systems. In this study, PB-treated group II showed a decrease in the enzymatic activity by 60.06% with respect to the control, group I; RF-treated group III, by 25.73% of the dip in its activity. The combination-treated groups IV and V demonstrated an increase in its activity by 47.52% and 79.94% as compared to group II (Figure 3).

#### 3.3.2. Superoxide Dismutase (SOD)

It is also a main antioxidant enzyme in a biological system. Groups II and III exhibited a decrease in the enzymatic activity by 77.10% and 7.21% in comparison to the control, respectively. However, groups IV and V displayed enhancement in the activity by 121.05% and 187.79% concerning group II (Figure 3).

#### 3.3.3. Glutathione Reductase (GR)

Groups II and III demonstrated dip in the activity by 79.48% and 14.26% concerning the control while groups IV and V showed an increase in the activity by 232.03% and 309.37% as compared to group II (Figure 3).

#### 3.3.4. Reduced Glutathione (GSH)

It is a prominent cellular reductant. Groups II and III exhibited a decline of 69.85% and 11.26% as compared to group I while groups IV and V displayed replenishment in its level by 144.73% and 167.11% concerning group II (Figure 3).

### 3.4. Effect on Macromolecular Oxidation

#### 3.4.1. Total Carbonyl Content

In the present study, groups II and III demonstrated an enhancement in the carbonyl content by 151.67% and 26.53% with respect to the control. Groups IV and V showed a decrease in the level by 35.18% and 43.28% as compared to group II (Figure 4).

#### 3.4.2. Malondialdehyde Level (MDA Levels)

In the present investigation, groups II and III exhibited an increase in its level by 152.90% and 43.87%, while groups IV and V displayed a decrease in its level by 22.19% and 31.37%, respectively, in comparison to group II (Figure 4).

### 3.5. Assessment of Mode of Cell Death

#### 3.5.1. Evaluation of Apoptosis: Activity of Caspase-3

Caspase-3 is an important enzyme that is elevated during apoptosis induction and progression. Group II showed a dip in its activity by 72.44%. In comparison, group III demonstrated an increase in its activity by 13.84% as compared to the control. Groups IV and V exhibited an elevation in its activity by 139.75% and 208.95% concerning group II, respectively (Figure 5).

#### 3.5.2. Assessment of Necrosis by the Activity of Lactate Dehydrogenase (LDH)

LDH is one of the significant indicators for necrotic progression in the living system [25]. In the present investigation, group II showed an increase in its activity by 405.10% while group III displayed a decline in its activity by 149.19% in comparison to the control, group I. Among the combination groups, groups IV and V demonstrated a decrease in its activity by 36.41% and 47.28%, respectively, as compared to group II (Figure 5).

### 3.6. Assessment of Damage on Nuclear DNA by Comet Assay

This assay is a reliable technique for the assessment of toxic abuse on nuclear DNA in the target tissues. In the present study, a comet assay was conducted on the liver tissues from the treated animals in which groups II and III showed an increase in the tail length by 100.92% and 23.06% concerning the control, group II. However, the combination groups VI and V demonstrated a decrease in the tail length by 17.38% and 30.79%, respectively, as compared to group II (Figure 6).

### 3.7. Histological Evaluation

Histopathological examination of the liver tissues from control rats (group I) showed typical hepatic architecture. The cytoplasm of their hepatocytes was normally distributed with normal regular nuclei beside the usual central vein and the blood sinusoids with Kupffer cells equally distributed into the hepatic lobule (Figure 7(a), Table 1). However, histological examination of many sections of PB-treated (group II) rats demonstrated extensive damage in their hepatic tissues (Figure 7(b), Table 1) as compared to the normal rats (group I). The hepatocytes had altered cytoplasm characterized by coarse, pink, and darkly stained granules and numerous vacuoles. A dilated central vein, abnormal vesiculation, and irregular shape of nuclei were vivid signs of histological alteration in comparison to the control. Besides, these tissues showed vast infiltration of inflammatory cells into hepatic tissues, especially around the central vein as a significant histopathological marker (Figure 7(b)). Moreover, different types of leukocytes could be recognized, especially neutrophils. However, some inflammatory cells with mild alterations were observed in the sections of group IV (PB-challenged rats treated with vitamin B_2_ at the dose of 2 mg/kg) (Figure 7(c), Table 1). The hepatic architecture in this group was found to be improved in comparison to group II rats. Furthermore, PB-challenged rats treated with vitamin B_2_ at a dose of 4 mg/kg (group V) demonstrated significant improvement in their hepatic tissue amounting close to the control section. Besides, there was a minimal number of inflammatory cells with relatively big and abundant Kupffer's cells in group V sections (Figure 7(d), Table 1). Besides, the hepatocytes appeared more or less normal in size and shape, yet their cytoplasm stained darker with eosin. Also, the cytoplasmic vacuoles were less in number, and the nuclei of most of the hepatocytes seemed normal.

## 4. Discussion

A great deal of literature has confirmed that RF has an excellent antioxidant property that can be taped to nullify the toxic effects of many xenobiotics and drugs [14, 27, 29, 30]. PB-induced toxicities because of its extensive usage in edibles, drinking water, colas, paints, and cosmetics are one of the profound clinical challenges in society. The present study is aimed at investigating if the administration of RF can alleviate PB-induced toxic insults in vivo. The research entails that the vitamin shows excellent antioxidant property blunting the PB-induced toxicities in vivo evidenced by enhanced activity of key antioxidant enzymes and protein as well as a decrease in the prominent toxicity and liver function markers significantly. Besides, the vitamin triggered apoptosis in the PB-induced damage in the cells of the liver besides containing the necrosis in the same (Figure 8). The comet assay and histopathological analysis further validated the trend of the undertaken parameters in the current work.

It is already well known that PB exerts the toxic insults in vivo during its biotransformation by generating reactive oxygen species that exacerbate the cellular redox balance and structural integrity in the target tissues [7, 31]. PB, being a strong oxidant, elicits ROS leading to extensive lipid peroxidation and depression in the level of GSH [7, 32, 33]. These aggressive radicals further invade the cell membrane and membraned organelles (mitochondria, lysosome, Golgi bodies, and endoplasmic reticulum) of the target cells. Also, they affect the biological activity of macromolecules (proteins, enzymes, lipids, and carbohydrate) that consequently leads to extensive tissue damage and cellular dysfunction [34, 35]. Many studies entail that PB hence causes extensive necrosis and apoptosis as consequences of a high dose or after accumulation for an extended duration in the biological system [16]. In addition, the biotransformed versions of PB generate hyperactive metabolites (bromate and bromide radicals) that are very invasive to cellular macromolecules and structure [36, 37]. Furthermore, PB-induced ROS and NOS have been reported to cause chromosomal aberration, DNA adduct formation, and generation of 8-OH dG after oxidative damage to DNA [32, 34]. Hence, the compound directly or indirectly (by its generated ROS) interfere or compromise the biological efficacy of many of the critical proteins and allied macromolecules disrupting many of the cellular functions ([38]a). All these cellular events consequently implicate the mutagenic and carcinogenic potentials of PB during its overdose or extended stay in the biological system [39, 40]. The results also show hepatotoxicity of PB prominently by elevating oxidative stress and affecting the essential macromolecules as well as distortion of structural components of the target cells. The current findings are in accord with the previous work published by Bayomy et al. [16].

On the other hand, the vitamin, RF, acts as a natural antioxidant alone or as a component of major antioxidant enzymes like reduced glutathione (GSH), glutathione reductase (GR), and glutathione peroxidase (GPx) [41]. The vitamin is an excellent free radical scavenger that can neutralize the aggression of the free radicals (ROS, RNS) because of the presence of an isoalloxazine ring in its structure [42]. It is the reason behind replenishment in these antioxidant parameters after administration of RF in the treatment (PB-administered) groups III to V in the present work. Earlier, Liang et al. [43] have reported that deficiency of RF not only causes depletion of GSH and SOD activity but also causes elevated lipid peroxidation. In our study, the reverse trend is evident upon RF supplementation to the PB-treated rats. Some of the studies also indicate that RF can enhance the specific activity of key antioxidant enzymes, including SOD, GPx, and CAT [42, 44], and the present findings are also in the same agreement. It is also documented that RF, if administered in a moderate amount in vivo, can trigger an extrinsic pathway of apoptosis. In contrast, it triggers intrinsic pathways along with extrinsic as well as ubiquitin/proteasome pathway if it is taken in a higher amount [45]. Besides, the vitamin has been reported to downregulate many antiapoptotic factors (P13 K, JNK, and ERK K phosphorylation) and also upregulate many proapoptotic factors (cytochrome C, Smac/Diablo, and htr A2/Omi). Interestingly, its anti-inflammatory and antipain properties make it highly recommendable for effective cancer treatment [45, 46]. In addition, various studies have deciphered that RF is a potent apoptosis-inducing molecule in diverse types of cell lines like HL-60 and HeLa under photoirradiation [47]. Earlier, Santos De Souza et al. [48] and De Souza Queiroz et al. [49] in separate studies on different cell lines reported induction of Fas-FasL-mediated apoptosis by RF under photoillumination. Recently, Khan et al. [30] have shown that the photoactivated vitamin caused cell death in mice with lung carcinoma.

It is noteworthy that the vitamin is a strong antioxidant in its native form, but it can also act as a prooxidant under photoillumination. Both of its properties are being exploited for medical intervention in various clinical challenges [30, 46]. Besides, its adequate supplementation improves the intestinal mucosa for the absorption of nutrients, enhancing the overall health of the individuals in the many studies [50]. In normal conditions, RF is absorbed as much as the body requires it. Still, in stress conditions, it can accumulate in the mitochondria and trigger the release of cytochrome C paving the ways for apoptosis induction [51–53]. In the present study, administration of oxidant like PB causes stress condition that prompts RF to act as an antioxidant as well as a free radical scavenger. This action of RF firstly absorbs the toxic shock of PB in a dose-dependent manner by elevating the activity of major antioxidant enzymes and GSH. In addition, RF can bring down the oxidative stress level and proportionate the ATP level (by enhancing intestinal mucosa absorption and boosting metabolism) that helps the partially damaged cells to undergo a normal cell cycle; at the same time, such concurrent conditions also trigger programmed cell death in the damaged cells [25, 27, 29, 38, 54, 55]. The study clearly shows that PB triggers more necrotic and inflammatory features besides apoptosis. At the same time, RF favors apoptosis, ceasing necrosis, and inflammation, as evidenced by the pattern of caspase-3 and LDH activity. Further, the comet assay and histopathological analysis confirm these results. The longer tail length shown by PB (group II) indicates the occurrence of necrosis. In contrast, the large fan-like tails with small heads (hedgehogs) in the combination groups (IV and V) endorse apoptosis in the damaged target cells [56]. The present investigation, hence, postulates the putative mechanism action of the alleviative effect of RF against PB-induced hepatotoxicity (Figure 8). However, further study is warranted to discourse the in-depth mechanism.

## 5. Conclusion

RF (vitamin B_2_) counters the PB-induced oxidative stress and restores cellular functions by replenishment of the GSH level and activity of key antioxidant enzymes concomitant with lowering the lipid and protein peroxidation in the target cells. Also, the vitamin protects PB-induced hepatotoxicity by promoting healing of the partially damaged cells as well as triggering apoptosis in the extensively damaged cells.

## Figures and Tables

**Figure 1:** Bar graph showing the level of liver function tests—alkaline phosphatase (ALP), aspartate transaminase (AST), and alanine transaminase (ALT)—in the serum samples. All data has been expressed in the mean ± SD of six independent experiments. The marks “a, b, and c” were used as asterisk marks to show significance difference from the negative control (CN^−^, group I) at *p* less than 0.05, 0.005, and 0.001 while the marks “x, y, and z” were used as asterisk marks to show significance difference from the positive control (CN^+^, group II) at *p* less than 0.05, 0.005, and 0.001.

**Figure 2:** Bar graph showing the level of liver toxicity markers—gamma glutamyl transferase (GGT), glutathione-S-transferase (GST), and thioredoxin reductase (TR)—in the liver samples. All data has been expressed in the mean ± SD of six independent experiments. The marks “a, b, and c” were used as asterisk marks to show significance difference from the negative control (CN^−^, group I) at *p* less than 0.05, 0.005, and 0.001 while the marks “x, y, and z” were used as asterisk marks to show significance difference from the positive control (CN^+^, group II) at *p* less than 0.05, 0.005, and 0.001.

**Figure 3:** Bar graphs showing the activity of key antioxidant parameters—superoxide dismutase (SOD), catalase (CAT), glutathione reductase (GR), and glutathione (GSH)—of various treatment groups. All data has been expressed in the mean ± SD of six independent experiments. The marks “a, b, and c” were used as asterisk marks to show significance difference from the negative control (CN^−^, group I) at *p* less than 0.05, 0.005, and 0.001 while the marks “x, y, and z” were used as asterisk marks to show significance difference from the positive control (CN^+^, group II) at *p* less than 0.05, 0.005, and 0.001.

**Figure 4:** Bar graphs showing the level of carbonyl content and malondialdehyde (MDA) in the liver samples of indicated animal groups. All data has been expressed in the mean ± SD of six independent experiments. The marks “a, b, and c” were used as asterisk marks to show significance difference from the negative control (CN^−^, group I) at *p* less than 0.05, 0.005, and 0.001 while the marks “x, y, and z” were used as asterisk marks to show significance difference from the positive control (CN^+^, group II) at *p* less than 0.05, 0.005, and 0.001.

**Figure 5:** Bar graphs showing the activity of caspase-3 and lactate dehydrogenase (LDH) in the liver samples of indicated animal groups. All data has been expressed in the mean ± SD of six independent experiments. The marks “a, b, and c” were used as asterisk marks to show significance difference from the negative control (CN^−^, group I) at *p* less than 0.05, 0.005, and 0.001 while the marks “x, y, and z” were used as asterisk marks to show significance difference from the positive control (CN^+^, group II) at *p* less than 0.05, 0.005, and 0.001.

**Figure 6:** Showing the average picture of the comet of the liver cells of indicated animal groups. All data of the comet tail length has been expressed in mean ± SD. “a, b, and c” were used as asterisk marks to show significance difference from the negative control (CN^−^, group I) at *p* less than 0.05, 0.005, and 0.001 while “x, y, and z” were used as asterisk marks to show significance difference from positive control (CN^+^, group II) at *p* less than 0.05, 0.005, and 0.001.

**Figure 7:** Representative photomicrographs showing the liver tissue section from (a) control without any treatment (group I), (b) riboflavin-supplemented group (group III), (c, d) PB-challenged group (group II), (e, f) PB-challenged and treated with riboflavin at the dose of 2 mg/kg group (group IV), and (g, h) PB-challenged and treated with riboflavin at the dose of 4 mg/kg group (group V). Examined sections show that PB induced severe damage to the hepatic tissue pattern. Narrow blood sinusoids (green arrows) with vacuolated hepatocytes (red arrows) were remarkably observed. The liver tissues were infiltrated with inflammatory cells (yellow arrows), especially around the central vein, which was found with severe dilatation in comparison with the control one. A marked improvement was observed in PB-challenged rats treated with riboflavin (group IV) (e, f). This improvement was dose-dependent since 4 mg of riboflavin (g, h) was found to remarkably restore a hepatic pattern close to that of the control liver tissue. All rat sections were stained with H&E and photographed at a magnification of ×400.

**Figure 8:** Depiction of the putative mechanism involved in the ameliorative efficacy of RF against PB-induced toxicities, indicating critical events in the target cells.

**Table 1:** A rating between − (no change) and +++ (severe damage) of the histopathological alterations into the hepatic tissues. The score was assigned for each investigated section of all the groups. Sections from at least five rats were carefully investigated.

Treatment groups	Control (group I)	Potassium bromate (group II)	Riboflavin (group III)	Potassium bromate+riboflavin dose I (group IV)	Potassium bromate+riboflavin dose II (group V)
Dilated central vein	(−)	(+++)	(−)	(++)	(+)
Abundance of Kupffer cells	(−)	(+)	(−)	(++)	(+++)
Vacuolated hepatocyte cytoplasm	(−)	(+++)	(+)	(++)	(−)
Hyaline and eosinophilic hepatocyte cytoplasm	(−)	(−)	(−)	(−)	(+)
Degenerated hepatocyte nuclei	(−)	(+++)	(−)	(++)	(+)
Unclear boundaries of hepatocytes	(-)	(++)	(+)	(++)	(+)
Hemolysed blood	(−)	(+)	(−)	(+)	(−)
Narrow sinusoids	(−)	(+++)	(+)	(++)	(+)
Infiltrated tissue with inflammatory cells	(−)	(+++)	(+)	(++)	(+)

## Data Availability

The data used to support the findings of this study are included in the article.
